# Synthesis of Ag@AgCl/CA and Visible-Light Photocatalytic Degradation of Oxtetracycline

**DOI:** 10.1155/2022/8466272

**Published:** 2022-08-21

**Authors:** Daxiang Gao, Hetong Yang, Zhen Shu

**Affiliations:** ^1^Jiangsu Vocational College of Agriculture and Forestry, Jiangsu, Jurong 212400, Singapore; ^2^Anhui Xuchen Biotechnology Co., Ltd, Anhui, Bengbu 233000, China

## Abstract

Chemical coupling, in-situ deposition of supported AgCl, and photoreduction were used to create Ag@AgCl/CA. The morphology, structure, and surface area of the prepared Ag@AgCl/CA were characterized by SEM, TEM, FT-IR, and BET. The photogenerated electron transport efficiency and visible light absorption were analyzed by photocurrent and electrochemical impedance spectroscopy (EIS), respectively. The surface electrical properties and degradation stability were evaluated by zeta potential measurement and cyclic catalytic degradation experiments, and the photocatalytic mechanism was proposed in detail based on the ESR test and trapping experiment. The results showed that the cluster of Ag@AgCl nanoparticles were distributed on the CA crosslinking structure. The prepared Ag@ AgCl/CA photocatalytic material has a high Zeta potential, stable photocurrent, and small photogenerated electron transfer resistance. It has good adsorption and photocatalytic degradation stability for OTC. The material has a relatively strong absorption in the visible light range. Temperature and initial pH had significant effects on the degradation of OTC by photocatalytic materials. The photocatalytic degradation rate was the highest at 40°C and pH6, and the photocatalytic degradation process conformed to the quasi-first-order reaction kinetics. Holes (h^+^) and superoxide radicals (·O_2_－) were the main active species for the degradation of OTC.

## 1. Introduction

In recent decades, antibiotics have been widely used in drug treatment and animal husbandry, and the potential harm caused by this has also attracted more and more attention. Tetracyclines (TCs) are one of the most widely used antibiotics [1, 2], which are widely used in drug treatment and animal husbandry. A large amount of antibiotic waste is discharged into the water, which can easily cause drug residues in the environment. Oxytetracycline (OTC), also known as oxytetracycline, is one of the tetracycline antibiotics. Due to its stable characteristics, OTC is difficult to decompose, resulting in environmental pollution. Biological treatment and physical adsorption of conventional sewage cannot be completely removed [3, 4]. For the use of chlorine gas or ozone for chemical oxidation and the Fenton process [5, 6], OTC can be oxidized, which often brings by-products and weak mineralization, harsh reaction conditions, and the need to work with other chemical reagents.

As a new technology, photocatalytic oxidation technology has a strong degradation effect on tetracycline antibiotic wastewater [7]. However, the efficiency of direct photocatalytic degradation is low, and its main tetracyclic structure is difficult to destroy, which will generate more hazardous intermediate products. Therefore, it is particularly important to study a photocatalyst for the degradation of tetracycline in the environment. At present, TiO_2_ is mostly used as a photocatalyst and its composite photocatalytic materials for the degradation of oxytetracycline [8, 9]. Recently, as a new type of visible light catalytic material, Ag@AgCl has attracted wide attention [10, 11]. Ag@AgCl refers to the monoplasmic Ag^0^ decomposed by the AgCl under light conditions that are loaded on the surface of AgCl. The Ag^0^ has a surface plasmon resonance (SPR) effect, good conductivity, and electron storage performance, which can enhance the absorption of visible light by catalytic materials, promote the transmission of electrons, and contribute to the separation of photogenerated electron-hole pairs. However, the poor adsorption capacity, easy agglomeration, and subsequent complex solid-liquid separation of pure Ag@AgCl also limit the application of powdered Ag@AgCl nanocomposites. Loading Ag@AgCl nanocomposites on the surface of porous materials can effectively solve the problems of nanoparticle agglomeration, weak adsorption capacity, and difficult separation and recovery while retaining high catalytic activity [12–14]. Sodium alginate (SA) is a kind of natural polysaccharide, that is stable, safe, nontoxic, and easy to obtain. It chelates with Ca^2+^ to form calcium alginate gel with a three-dimensional network structure, which can well adsorb heavy metals, azo dyes, organic acids, and other complex pollutants. There were many studies, while the combination of catalytic degradation materials and calcium alginate gel was less studied, which is the focus of the future. The composite photocatalyst of Ag@AgCl and calcium alginate (CA) gel for the degradation of OTC is rarely reported.

In this study, a stable microgel was prepared by the dispersion of cationic emulsifier cetyltrimethylammonium bromide (CTAB). The microgel was loaded with AgCl by ion exchange and in-situ deposition methods, and then part of AgCl was reduced to the Ag nanoparticles by photoreduction reaction and dispersed on the surface of AgCl. This material, Ag@AgCl/CA, is composed of a small particle with a strong adsorption capacity, a short photocatalytic degradation time, a high catalytic efficiency, a wide response range of visible light waves, and easy recycling, which can be used for the degradation of actual pollutant wastewater.

## 2. Materials and Methods

### 2.1. Materials

CTAB, SA, Ca(NO_3_)_2_AgNO_3_, NaCl, and OTC(AR, Xilong Chemical Co.). Tert-butanol (TBA), ethylenediaminetetraacetic salt (EDTA-2Na), and phenylquinone (p-BQ) (AR, West Asia Chemical Technology Co., Ltd., Shandong). All the water used in the test was deionized water.

### 2.2. Preparation of Ag/AgCl @CA

After ultrasonic dispersion for 30 min, 10 g/L of 16 mL of CTAB solution was added to 2 g/L of 100 mL of SA solution, and then CTAB and SA solution were fully mixed. Under magnetic stirring, 12 mL of 50 g/L AgNO_3_ solution was slowly added, and after 15 min of magnetic stirring, 40 mL of 20 g/L (CaNO_3_)_2_ solution was slowly added to the mixed suspension. After continuing stirring for 15 min, 10 mL of 20 g/L NaCl solution was added slowly and dropped. Stirring was closed after 30 min, and the mixed system stood for 24 h. The particle precipitate was obtained by filtering through double-layer gauze and washed with deionized water 5 times. Then the precipitate was added into a 250 mL flask containing 50 mL of deionized water and irradiated for 30 min by using a 10 W UV lamp under magnetic stirring. Ag@AgCl/CA was obtained through double-layer gauze filtration and vacuum freeze-dried.

### 2.3. Characterizations of Photocatalytic Materials

The morphologies were collected with a field emission scanning electron microscope (SEM) (Quattro S, FEI, USA). The microstructures were examined by a transmission electron microscope (TEM) (JEM-2100, Japan Electronics Co., Ltd), with an acceleration voltage of 200 kV. The chemical bonding status of the samples was analyzed on an FT-IR spectrometer (IRtracer-100, Shimadzu, Japan), with a resolution of 4 cm^−1^ and a scanning range of 400–4000 cm^−1^. The Raman spectra of the samples were measured with a laser confocal Raman spectrometer (LabRAM HR Evolution, HORIBA, France). The specific surface area of the samples was calculated by using an automatic specific surface area analyzer (BELSORP-max, MicrotracBEL, Japan). The zeta potential of the samples was measured by a zeta potentiometer (ZEN3600, Malvern, UK). The UV-visible absorbance spectra of the samples were obtained by using a UV-visible spectrophotometer (lambda750, PerkinElmer, America). The photocurrent and electrochemical impedance spectroscopy (EIS) of the composite were tested by an electrochemical workstation (CHI-660E, Chenhua, Shanghai) with a Na_2_SO_4_ solution of 0.05 mol L^−1^. The UV-visible absorbance spectra of the degradation solution were obtained by means of a UV-visible spectrophotometer (UV-2600, Shimadzu, Japan). The electron spin resonance (ESR) spectra in the solution were detected under dark or visible light (*λ* > 420 nm) with an electron paramagnetic resonance spectrometer (JES-FA200, Japan Electronics Co., Ltd).

0.2 g of the prepared Ag@AgCl/CA was added into a 100 mL triangular flask, and then 60 mL of 10 mg/L OTC solution was added. After mixing, the initial pH value was adjusted to 6.0, and the temperature was controlled at 40°C. After magnetic stirring for 30 min in the dark, the triangular flask was placed under a 300 W xenon lamp (*λ* > 420 nm), and the distance between the light source and the liquid level was about 5 cm. The time was started under magnetic stirring, and 3 mL of the upper reaction solution was taken out every 2 min as the test solution. The absorbance change was measured to evaluate the degradation activity of the catalytic material. The relationship curve between the *C*_t_/*C*_0_ of the OTC solution and the degradation time *t* in the degradation process is the photo-degradation curve, where *C*_0_ and *C*_t_ are the OTC concentrations (mg/L) at reaction times 0 and t, respectively. The Ag@AgCl/CA was recovered, washed with deionized water, repeated photocatalytic experiments, and recycled for five cycles.

By integrating the Langmuir-Hinshelwood (L-H) kinetic equation, the first-order reaction rate equation was obtained to investigate the kinetic relationship of the prepared photocatalytic material: ln (*C*_0_/*C*_t_) = *kt* + *A*, where *k* was the first-order apparent rate constant, *C*_0_ was the OTC concentration (mg/L) after the adsorption equilibrium of OTC, and *C*_t_ was the OTC concentration (mg/L) at *t* irradiation time(min).

In order to better understand the active radicals that play a major role in the photocatalytic degradation of OTC, radical trapping experiments were performed. In the experiment, TBA (5 mL), EDTA-2Na (0.5 g), and p-BQ (0.5 g) were used as capture agents for O_2_－、·OH, and h^+^, respectively, and (C_0_-C_t_)/C_0_ was used to indicate the photocatalytic degradation rate (%) of OTC at *t* time (min).

## 3. Results and Discussion

### 3.1. Structural Analysis of the Material

Figures 1 and 2 show the SEM image and TEM image of the Ag@AgCl/CA composites, respectively. A large number of irregular Ag@AgCl particles were successfully loaded onto the gel structure of calcium alginate (CA), partially overlapped, and stacked in clusters. Ag@AgCl particles are spherical with an uneven particle size of 50–100 nm. It can be seen that the Ag@AgCl particles were successfully loaded into the Ca^2+^ crosslinking gap. The gel grid structure can act as a separator to effectively segment the cluster Ag@AgCl particles, which is beneficial to the adsorption and rapid degradation of OTC by the composites to a certain extent and effectively improve the photocatalytic performance of the composites.

Figures 3 and 4 show the EDS spectra and the surface scanning distribution of the main elements of the composites, respectively. The results showed that the samples contained Ag, Cl, C, O, N, Ca, Br, and other elements. The mass concentration of the Ag element was higher than that of the C element, and the concentration of the Ag atom was also higher than that of C and O, while the concentration of the Cl atom was about half of that of the Ag atom, namely, Ag: AgCl = 1 : 1, indicating that each AgCl particle surface was roughly adhered by Ag nanoparticles (AgNPs). In addition, the materials contain certain N and Br atoms, indicating that the prepared catalytic materials contain a small amount of AgBr particles and CTAB cationic components, and a small amount of AgBr particles can also cooperate with Ag@AgCl for the catalytic degradation of pollutants. The Ag@AgCl particles dispersed on CA gel could effectively enhance the adsorption performance and catalytic degradation performance of the composite.

### 3.2. FT-IR Analysis

According to Figure 5, the absorption peak at 1030 cm^−1^ in the composite Ag@AgCl/CA belongs to the C-O-C stretching vibration absorption peak of the epoxy group[15]. The peaks at 1597 cm^−1^ and 1403 cm^−1^ are mainly attributed to the expansion vibration of C = O(-COOH) and the bending vibration peak of -OH (-COOH) in SA, respectively. The absorption peak at 2915 cm^−1^ is attributed to the stretching vibration of methyl (-CH_3_), and the absorption peak at 2851 cm^−1^ may be caused by the stretching vibration of methylene (-CH_2_^−^) in the alkyl chain of CTAB. It is known that the vibration peak of free hydroxyl is located at 3640∼3610 cm^−1^, while the stretching vibration peak of associated hydroxyl exists at 3400∼3200 cm^−1^. Therefore, the composite material has a strong peak absorption peak near 3375 cm^−1^, which is the expansion vibration peak of the associated hydroxyl group(-OH).

### 3.3. Adsorption Property Analysis

The specific surface area and pore structure of the adsorbent determine the adsorption effect. Usually, in the adsorption process, the larger the specific surface area of the material, the stronger the adsorption performance of the material is [16].  Figure 6 shows the N_2_ adsorption-desorption isotherm and pore size distribution of the Ag@AgCl/CA. The isotherm complies with the IV-type, indicating that the composite has a mesoporous structure, which is conducive to the contact between the catalyst and OTC, the absorption of visible light, the reduction of electron-hole recombination, and the improvement of the photocatalytic degradation performance of the composite [17]. The specific surface area and average pore size of the material are 0.96553 m^2^/g and 21.311 nm, respectively, and the pore size distribution is between 2 and 100 nm. According to the photocatalytic oxidation mechanism, the recombination of photogenerated electrons and holes on the catalyst surface is completed within 10^−9^ s, but the carrier capture rate is relatively slow, which usually takes 10^−8^～10^−7^ s. Therefore, only the pollutants adsorbed on the catalyst surface are likely to obtain highly active electrons and holes for the reaction [18].

### 3.4. Photocurrent and EIS

Efficient charge transfer and separation are important factors affecting photocatalysis.  Figure 7 shows the transient photocurrent response properties of Ag@AgCl/CA under each opening and shading light. The Ag@AgCl/CA could generate a fast and stable photocurrent with good reversibility under visible light. Therefore, this catalytic material has strong photosensitivity, good photocurrent response, high photogenerated electron transfer efficiency, and photogenerated electron-hole pair separation efficiency, indicating that the prepared material has high photocatalytic activity.

Electrochemical impedance spectroscopy (EIS) is an effective method to analyze the interface charge transfer of a photocatalyst. The smaller the arc radius in the EIS, the higher the electron-hole separation efficiency of the material [19].  Figure 8 shows that the arc radius without light is significantly larger than that with light. Therefore, under light radiation, the Ag@AgCl/CA has lower photogenerated electron transfer resistance and lower electron-hole recombination, showing good photocatalytic performance.

### 3.5. Electrical Property

The zeta (*ζ*) potential is an important indicator to characterize the stability of colloidal dispersion system. The higher the absolute value of Zeta potential is, the more stable the dispersion system is [20].  Figure 8 shows that the Zeta potential of pH 4, 5, 6, 7, and 8 is −30.1 mV, −32.7 mV, −34.8 mV, −30.9 mV, and −43.5 mV, respectively, indicating that the catalytic material has a negative charge at pH4～8. At this time, there is a repulsion between the catalytic material particles, resulting in a steric effect, indicating that the catalytic material has strong stability.

In addition, the study showed that when the initial pH of the solution was greater than 7, Ag^+^ would combine with the hydroxide in the solution to form precipitation, which caused the solution to change color. Therefore, the catalyst was used well under acidic conditions.

### 3.6. UV-Vis DRS Characterization

It can be seen from Figure 9 that the Ag@AgCl/CA catalytic material not only has strong absorption in the ultraviolet region below 380 nm but also has strong absorption in the visible region of 450∼650 nm. It is reported that the indirect band gap of AgCl is about 3.25 eV. In addition to the ultraviolet absorption band, AgCl has almost no absorption performance in the range of 400∼800 nm [21]. Therefore, the catalytic material has a strong absorption performance in the visible region, which should be attributed to the resonant absorption band generated by the SPR effect of the Ag nanoparticles [22]. Compared with Ag@AgCl, the visible light absorption of the material is significantly enhanced.

### 3.7. Photocatalytic Degradation Performance

#### 3.7.1. Effect of the Temperature

Figure 10 shows the absorption curve of OTC photocatalytic degradation at 40°C for different times. OTC has two obvious absorption peaks at 275 nm and 355 nm, respectively. After 30 min of dark adsorption, the absorption peaks were significantly reduced, and the absorption peak at 275 nm disappeared after 6 min of irradiation, while the absorption peak at 355 nm was significantly weakened. With the extension of irradiation time, the absorbance at 355 nm decreased gradually, and the absorption peak showed a blue shift.

Figures 11(a) and 11(b) show the degradation curves and the fitted kinetic curves for the photocatalytic degradation of the OTC. At different temperatures, the relationship between ln (*C*_0_/*C*_t_) and *t* has good linearity, which conforms to the first-order kinetic model of photocatalytic degradation. An appropriate increase in temperature could promote the degradation of OTC because a suitable increase in temperature is conducive to the adsorption of OTC and could promote the thermal movement of molecules to accelerate the reaction. The degradation rate of OTC was the highest at 40°C. After 18 min of irradiation, the photocatalytic degradation rate of OTC reached 84%, indicating that the prepared Ag@AgCl/CA had an excellent photocatalytic degradation effect on OTC.

#### 3.7.2. Effect of the Initial pH Value

The initial pH is also one of the important parameters affecting the chemical reaction.  Figure 12 is the photocatalytic degradation absorption curve of the OTC solution at initial pH6. In general, the effect of pH on photodegradation is mainly due to the change of proton state and absorption peak of organics [23]. Under different pH, OTC shows different ion forms (OTC ^+^, OTC, OTC^−^) [24]. Since the prepared Ag@AgCl/CA has a negative charge in pH 4∼8, and OTC gets a H^+^ and is positively charged under acid conditions [25]. Therefore, it has a strong adsorption capacity on OTC under acid conditions, which further promotes the photodegradation efficiency of OTC.  Figure 13 shows that the photocatalytic degradation of the OTC conforms to the first-order reaction kinetics at different pH, and the *k* (0.10607 min^−1^) is the highest at pH 6.

### 3.8. Stability Test

In practical applications, the stability and reliability of photocatalysts are particularly important. The activity of the photocatalytic material had not changed significantly after 5 times of recycling (Figure 14), and the degradation rate of OTC was still more than 95.0%, indicating that the Ag@AgCl/CA has good photocatalytic stability and reusability. As a visible light catalyst, it has great potential in practical production.

### 3.9. Photocatalytic Mechanism Analysis

Figure 15 shows the ESR spectrometer of ·O_2_^－^and ·OH. The signals of DMPO-·OH and DMPO-·O_2_^－^were not detected in the system in the dark. However, the characteristic quadruple peaks of DMPO-·O_2_^－^and DMPO-·OH could be clearly observed after 5 and 10 min of visible light.  Figure 15(a) shows the characteristic signal peak intensity ratio (1 : 1:1 : 1) of DMPO-·O_2_^－^, with the hyperfine splitting constant values(*α*_*N*_ = 1.337 mT, *α*_H_*β* = 1.025 mT) and spectral splitting factor *g* (2.0007).  Figure 15(b) displays the characteristic peak signal intensity ratio (1 : 2:2 : 1) of DMPO -·OH with the hyperfine splitting constant values (*α*_*N*_ = *α*_H_^*β*^ = 1.500 mT) and spectral splitting factor *g* (2.0008). With the increase in irradiation time, the peak intensities of DMPO-·OH and DMPO-·O_2_^－^increased gradually. The results indicate that ·OH and ·O_2_^－^appear under light conditions, and light irradiation is a necessary condition to stimulate active substances.

The free radical capture experiments were carried out in order to better understand the actives that play a major role in the photocatalytic degradation of OTC by the Ag@AgCl/CA.  Figure 16 shows the photocatalytic degradation rate and fitting kinetics of OTC with and without different scavengers. The degradation rate of OTC was 99% after 18 min without scavengers. As a ·O_2_^－^scavenger, the addition of p-BQ greatly reduced the degradation rate, and only 5.6% of OTC was degraded, which indicated that a large amount of ·O_2_^－^ was generated, and ·O_2_^－^was a main reactive active species. The addition of EDTA-2Na reduced the degradation rate to 48.4%, while the addition of TBA had little effect. The above results indicate that ·O_2_^－^plays a leading role, followed by h^+^, and ·OH does not, during the photocatalytic degradation of OTC.

Under visible light irradiation, AgNPs on the surface of the Ag@AgCl/CA composites were excited by the SPR effect, resulting in e^−^and h^+^. Because the Fermi level of the AgNPs is relatively low compared with the conduction band phase of AgCl, and because the existence of Cl^−^ on the surface of AgCl makes the surface of AgCl negatively charged, resulting in a polarization effect, the generated e^−^ was rapidly transferred from the Ag@AgCl interface to the surface of AgNPs, and captured by dissolved oxygen in the water to form reactive ·O_2_^－^, which further decomposed OTC. At the same time, the photogenerated h^+^ was transferred to the surface of AgCl, and h^+^ itself has strong oxidation, which could effectively degrade OTC. In addition, the h^+^ transferred could also react with Cl^−^ to generate Cl^0^ free radicals. Cl^0^ could also rapidly oxidize the OTC adsorbed on the surface of the catalyst, and then Cl^0^ was reduced to Cl^−^ [26]. In addition, the material has a gel grid structure, large pore size structure, and specific surface area, as well as more negative charges under acidic conditions, which is conducive to the adsorption of more OTC molecules and is also one of the reasons why the material has high visible light catalytic activity.

## 4. Conclusions

The insoluble particle photocatalytic material was prepared by the CA gel template loading Ag@AgCl, which has a simple process, large specific surface area, high adsorption performance, stable photocurrent, and strong absorption of visible light . The photocatalytic material has a good degradation effect on the OTC wastewater and has a high catalytic efficiency and short catalytic time. The catalytic material is composed of small particles and has good photocatalytic stability and reusability. It is also easy to recycle. As a visible light catalyst, it has great potential in practical production.

## Figures and Tables

**Figure 1:** The SEM of the sample.

**Figure 2:** The TEM of the sample.

**Figure 3:** The EDS profiles of the sample.

**Figure 4:** Electron diffraction pattern of the sample.

**Figure 5:** FT-IR spectra of the Ag@AgCl//CA.

**Figure 6:** (a) Adsortion-desorption isotherms and (b) pore size distribution of the Ag@AgCl/CA.

**Figure 7:** Transient photocurrent response (a) and electrochemical impedance spectra (b) of Ag@AgCl/CA.

**Figure 8:** Potential distribution.

**Figure 9:** UV-vis DRS of the Ag@AgCl/CA and Ag@AgCl.

**Figure 10:** The absorption curve of OTC photocatalytic degradation at 40°C.

**Figure 11:** (a) Degradation rates and (b) the fitted kinetic curves of OTC at different temperatures.

**Figure 12:** The absorption curve of OTC degradation at different initial pH.

**Figure 13:** (a) Degradation rates and (b) the fitted kinetic curves of OTC at different initial pH.

**Figure 14:** Stability test of OTC degradation.

**Figure 15:** ESR spectra of superoxide radical and hydroxyl radical: (a) ·O_2_^－^, (b) ·OH.

**Figure 16:** Effects of different scavengers on OTC degradation.

## Data Availability

The experimental data used to support the findings of this study are available from the corresponding authors upon request.
